The article "Protecting Endangered Species: Do the Main Legislative Tools Work?" was published in 2012. Journal: PLoS One.

# Protecting Endangered Species: Do the Main Legislative Tools Work?

**DOI:** 10.1371/journal.pone.0035730

**Published:** 2012-05-02

**Authors:** Katherine E. Gibbs, David J. Currie

**Affiliations:** Ottawa-Carleton Institute of Biology, University of Ottawa, Ottawa, Ontario, Canada; University of Veterinary Medicine Hanover, Germany

## Abstract

It is critical to assess the effectiveness of the tools used to protect endangered species. The main tools enabled under the U.S. Endangered Species Act (ESA) to promote species recovery are funding, recovery plan development and critical habitat designation. Earlier studies sometimes found that statistically significant effects of these tools could be detected, but they have not answered the question of whether the effects were large enough to be biologically meaningful. Here, we ask: how much does the recovery status of ESA-listed species improve with the application of these tools? We used species' staus reports to Congress from 1988 to 2006 to quantify two measures of recovery for 1179 species. We related these to the amount of federal funding, years with a recovery plan, years with critical habitat designation, the amount of peer-reviewed scientific information, and time listed. We found that change in recovery status of listed species was, at best, only very weakly related to any of these tools. Recovery was positively related to the number of years listed, years with a recovery plan, and funding, however, these tools combined explain <13% of the variation in recovery status among species. Earlier studies that reported significant effects of these tools did not focus on effect sizes; however, they are in fact similarly small. One must conclude either that these tools are not very effective in promoting species' recovery, or (as we suspect) that species recovery data are so poor that it is impossible to tell whether the tools are effective or not. It is critically important to assess the effectiveness of tools used to promote species recovery; it is therefore also critically important to obtain population status data that are adequate to that task.

## Introduction

For conservation efforts to succeed, it is critical to evaluate the effectiveness of available conservation tools and to adapt management accordingly [1]. The U.S. Endangered Species Act (ESA) is one of the oldest and most comprehensive pieces of endangered species legislation and one of the main mechanisms for preventing species' extinction [2], [3]. The main tools enabled under the act that are applicable to all species are protection from take, section 7 consultation, funding, recovery plan development and implementation, and critical habitat designation [4]. There are other tools such as Habitat Conservation Plans, Safe Harbor Agreements and Candidate Conservation Agreements that are used on a case by case basis [5].

However, even the main tools have not been applied equally to all species listed under the Act. This provides a quasi-experimental test of their efficacy: if the tools enabled under the ESA are effective, one would expect that, on average, recovery of species listed under the Act would be positively related to measures of the degree of implementation of those tools. Here, we ask: how strongly does the evidence support this prediction?

Our question is not whether *any* species have benefitted from the ESA; this is undoubtedly true: e.g. Aleutian Canadian goose, Robbins' cinquefoil and Kirtland's Warbler [6], [7]. Rather, we ask whether, on average, recovery is improved materially in species that have benefitted from the tools enabled under the ESA. Previous studies have concluded that various tools under the Act are effective, based on significant statistical relationships [8], [9], [10]. However, whether tools implemented under the ESA have had *detectable* effects (i.e., statistically significant) is at least partly an issue of statistical power. Arguably, the more important question is how large or small those effects have been. Extant work has not addressed this question.

Consider these tools in more detail. Once listed, species are protected from take, which includes harassing, harming, or killing [11]. Species also benefit from Section 7 consultation, which states that federal agencies must consult with the Fish and Wildlife Service (FWS) to ensure that their actions do not jeopardize the species [4]. The Fish and Wildlife Services and the National Oceanic Atmospheric Administration (NOAA) provide funding for a variety of purposes involving listed species [12], including habitat acquisition, research, and enforcement. Further, the Act requires that a recovery plan be developed and implemented for every listed species, except when such a plan will not promote conservation of the species [11]. The recovery plan details the conservation actions that are necessary for recovery. Critical habitat (CH), defined as the specific areas within the geographical area occupied by the species, at the time it is listed, essential to the conservation of the species, is designated at the time of listing when judged to be ‘prudent and determinable’ [11].

Critical habitat designation is the most controversial aspect of the Act [13]. Although required for all species, it is currently only in place for 43% of U.S. listed species [14]. Critical habitat can be cited as ‘undeterminable’ or ‘not prudent’ to avoid designation [15]. In early 2000, only 10% of species had CH designation. This prompted legal action, and a large number of designations were pushed through by court order [16], [17]. The Department of the Interior claimed that the flood of CH designations was undermining endangered species conservation by using up funds and that it “does not result in any benefit to the species that is not already afforded by the protections” in other aspects of the Act [18]. Federal agencies are already required under the Act to consult with FWS to ensure that their actions do not adversely modify species habitat to a point where it would jeopardize species [19]. However, this protection only applies to lands currently occupied by the species. Critical habitat designation can go a step further and designate areas that are currently unoccupied by the species but deemed necessary for their recovery [20]. This controversy highlights the necessity of studying the effect of CH designation on species recovery [4].

Earlier studies that have attempted to assess the effectiveness of the ESA yielded conflicting results. Kirkvliet and Langpap [8] examined the recovery status of 225 listed species and concluded that spending reduced the probability of species doing poorly but was unrelated to the probability of doing well. They found that having a recovery plan (either in progress or completed) decreased the probability of species being reported as declining and increased the probability of species being stable or increasing. They did not find evidence that CH designation promotes species recovery. Taylor et al. [10] considered a larger set of listed species (N = 1095). Looking separately at single species and multi-species recovery plans, they found a positive effect of single species recovery plans but no effect of multi-species plans. They argued that species with CH designation were more likely to be increasing and less likely to be decreasing than species without CH designation. In contrast, Male and Bean [9], using a similar data set that included federal funding, concluded that species status was positively related to funding but was not significantly related to CH designation. Miller et al. [21] calculated funding as the amount of money received divided by the amount requested in the species recovery plan. They found that with increased funding, species status was more likely to be improving. Boersma et al. [22] examined the effectiveness of recovery plans in detail and found that single species plans and those with a diversity of authors are related to increased likelihood of species doing well. In each case, the authors focus on whether statistical relationships are detectable, as opposed to how strong those relationships are.

In this study, we examine two measures of species recovery: population status trends (on which most earlier studies have focused) and the number of recovery objectives achieved (among those listed in the species' recovery plan). We test how much of the inter-specific variation in recovery of ESA-listed species can be statistically attributed to how long the species has been listed (i.e, the base protection from being listed), how long a recovery plan has been in place, whether and how long critical habitat has been designated, and federal funding. If such tools improve species' recovery, then change in species status over time and number of recovery objectives achieved should relate reasonably strongly to these variables. Since one of the main intentions of funding and recovery plan development is to support research and to increase what is known about a given species, we also look at the relationship between recovery status and the amount of published peer-reviewed scientific information available on each species. We look more closely at the effect of CH designation by comparing species' status before and after designation. We also test whether the effect of CH designation is stronger for species who are specifically threatened by habitat loss.

Not all species have a recovery status trend reported in each recovery report, presumably due to lack of information. We also test whether the availability of status information relates to the amount of peer-reviewed scientific information, funding, time listed, or taxonomic group.

## Methods

Recovery status was assessed for all U.S. and joint U.S./foreign species listed under the Endangered Species Act prior to 2003 (Dataset S1). Two measures of species recovery – change in population status over time, and the proportion of recovery objectives achieved by 2006, were extracted from biennial recovery reports to Congress from 1988–2006 [23]. Population status reports rate each species as decreasing, stable, increasing or unknown, relative to the previous report based on population size estimates as well as perceived threats [23]. These assessments are often based on qualitative information and can be based solely on the judgment of a species expert, but they are the best species status data available for all ESA listed species [22].

Using the population status data, we calculated an index of change in status over the period 1988–2006 following Male and Bean [19]. For a given species, we first assigned a value of −1, 0 or 1 to each status report for declining, stable or increasing, respectively. These values were then summed, resulting in a final species score ranging from −9 to +9. Not all species had a status report for every biennial period in the data set. For these species, we calculated the proportion of reporting periods for which the population trend was known. We adjusted the final status score by dividing it by the proportion of known reports such that all population trend indices are based effectively on an 18 year period. This assumes that missing status information is equal to the average of the observed reports. Our second metric of recovery status, the recovery objectives achieved, is reported on a scale from 1 to 4 representing the percent of recovery objectives that have been achieved, according to the most recent recovery report used in the analysis (2006). We excluded species with multiple listed populations where each population had a different status; otherwise they were included as one record. Species presumed extinct in the wild or found only in captivity were also excluded.

Yearly funding was obtained from annual expenditure reports to Congress covering 1989–2004 which include all reported federal and state funding [12]. For each species, we calculated mean yearly funding. Because different species require different amounts of funding, we also calculated mean yearly funding received as a proportion of the mean yearly estimated cost of recovery given in the recovery plan for each species [14]. Analysis using the proportional funding data is therefore limited to species that have a recovery plan with recovery cost estimates (739 species).

For each species, we recorded the number of years since listing, CH designation and recovery plan completion using 2004 as the base year [14]. Peer-reviewed scientific information was estimated as the number of studies found from a Web of Science search conducted in July 2007 of each species' scientific name. We also recorded whether habitat loss was a threat for each species, based on NatureServe [24] and the FWS recovery plans [14]. We separated threats into three categories: direct habitat loss (e.g. habitat destroyed for residential development), habitat related threats (e.g. habitat degradation, pollution) and non-habitat related threats (e.g. overharvest, predation or competition from introduced species). If any direct habitat loss threats were mentioned, then it was recorded as such regardless of whether other threats were also present. Species were grouped into seven taxonomic groups: amphibians, birds, fish, invertebrates, mammals, plants and reptiles.

Generalized linear models were used to test the relationships between measures of species recovery and the independent variables. General linear models were performed for the population status data and the proportion of periods for which a status estimate was available was used as a weighting factor. Proportional odds multinomial logistic models were performed for the recovery objective variable. We use McFadden's pseudo R-square as a measure of explained variability [25], [26]. We did these analyses for all species combined, and within taxonomic groups. Mean yearly funding and peer-reviewed information were log-transformed, and all variables were standardized (mean = 0, s.d. = 1).

We did two additional tests to focus more explicitly on the effect of CH designation. To determine whether the effect of CH designation on status depends on the degree to which species are jeopardized by habitat-related threats, we compared the effect of CH designation on status for each threat category separately. We did a second analysis using only species for which CH had been designated. This analysis included the 218 species with status information both before and after their CH designation. For these species, we calculated the difference between the average status before and after CH designation. To control for any positive effect of being listed, with or without CH, we also calculated the average change in status of species without CH designation.

## Results

This study included 1179 species listed before 2003, of which plants made up 61%, invertebrates 14%, fish 9%, birds 6%, mammals 5%, reptiles 3% and amphibians 2%. Population status data were available for 1146 species; 33 species were excluded because they had unknown status in every recovery report. We adjusted population status scores for a further 796 species that had at least one unknown status report. Considering all 1146 species, the trends in population status neither improved nor worsened from 1988–2006 (median slope = 0.0). The median status score for all species was −3: i.e., populations generally declined relative to earlier reports. Recovery objective data were available for 1169 species (all except 10 marine species under NOAA jurisdiction). Over all species, the median recovery objective value is a score of 1 which loosely corresponds to 0–25% of the recovery objectives achieved.

Recovery is detectably related to some of the factors expected to promote recovery, but the overall variation explained is small. In the strongest model, the proportion of recovery objectives achieved was significantly positively related to the number of years listed (p<0.0001; Fig. 1a), amount of peer-reviewed scientific information (p<0.0001; Fig. 1b), funding as a proportion of the amount required (p = 0.024), and years with a recovery plan (p = 0.005) (Table 1). A categorical variable distinguishing among taxonomic groups was also significant (p = 0.035): birds, mammals and fish have recovered better, on average, than plants, amphibians and invertebrates. The overall model explained 13% of the variation in recovery objectives achieved (i.e., pseudo R^2^ = 0.129).

**Figure 1:** Recovery objectives achieved as a function of years listed and scientific information. Scatter plots of recovery objectives achieved and (a) number of years listed and (b) amount of peer-reviewed scientific information. Peer-reviewed scientific information is calculated as the number of Web of Science search conducted in July of 2007 of each species' scientific name and is natural logarithm transformed. Lines on the graphs show LOWESS smoothing functions with tension = 0.7. N = 1169.

**Table 1:** Regression results for models relating ESA tools to species recovery.

Model	Dependent Variable	Independent Variable	Parameter estimate	P	Odds ratio	N	R^2^
**Model 1**	Proportion of recovery objectives achieved	Taxon	-*	0.035	-*	752	0.129
		Recovery plan	0.463	0.005	1.59		
		Critical habitat	0.063	0.476	1.07		
		Years listed	0.840	<0.0001	2.32		
		Scientific information	0.561	<0.0001	1.75		
		Proportional funding	0.249	0.024	1.28		
**Model 2**	Proportion of recovery objectives achieved	Taxon	-*	0.083	-*	1169	0.115
		Recovery plan	0.340	<0.0001	1.10		
		Critical habitat	0.075	0.227	1.08		
		Years listed	0.39	<0.0001	1.89		
		Mean yearly funding	0.431	<0.0001	1.54		
**Model 3**	Population status	Taxon	-*	0.017	-*	739	0.080
		Recovery plan	0.069	0.283	-		
		Critical habitat	0.038	0.302	-		
		Years listed	0.119	0.029	-		
		Scientific information	−0.016	0.724			
		Proportional funding	0.162	<0.0001	-		
**Model 4**	Population status	Taxon	-*	<0.0001	-*	1146	0.057
		Recovery plan	0.027	0.414	-		
		Critical habitat	0.025	0.394	-		
		Years listed	0.078	0.047	-		
		Mean yearly funding	−0.027	0.465	-		

General linear models were performed for the population status data and the proportion of periods for which a status estimate was available was used as a weighting factor. Proportional odds multinomial logistic models were performed for the recovery objective variable. We use McFadden's pseudo R-square for the multinomial models.

* *Taxon is a categorical variable and therefore the parameter estimates and odds ratios are given for each level and are not reported here. Significant variables appear in black text while non-significant variables appear in grey.*

We observed similar results for the change in population status over time. Status was significantly related to taxon (p = 0.017), years listed (p = 0.029) and proportional funding (p<0.0001; Fig. 2; pseudo R^2^ for full model = 0.080). Population status was also related to mean yearly funding, but less strongly than to proportional funding (Table 1). Peer-reviewed scientific information and mean yearly funding were strongly collinear (r = 0.635, p<0.0001; Fig. 3a); we therefore did not include both variables in our models.

**Figure 2:** Relationship between population status and funding. Scatter plot of species population status score and the proportion of funding requested in species recovery plan that has been received. Proportion of funding received is natural logarithm transformed. Line shows LOWESS smoothing function with tension = 0.7. N = 752.

**Figure 3:** Relationships between funding, scientific information and the proportion of known reports. Scatter plots showing the relationship between (a) mean yearly funding and the amount of peer-reviewed scientific information available on a species, (b) mean yearly funding and the proportion of known reports and (c) amount of peer-reviewed scientific information and the proportion of known reports. Peer-reviewed scientific information is calculated as the number of Web of Science search conducted in July of 2007 of each species' scientific name. Mean yearly funding and peer-reviewed scientific information are natural logarithm transformed. Lines on the graphs show LOWESS smoothing functions with tension = 0.7. N = 1169.

Within taxonomic groups, significant relationships were found for birds, fish, mammals, invertebrates and plants; however, once again, the effect sizes were quite small. Overall, years listed was the most important variable for all groups and peer-reviewed scientific information and funding were important for most groups. The strongest relationships (R^2^>0.15) were found for birds, mammals and plants. For birds, population status was significantly positively related to years listed (N = 69; pseudo R^2^ = 0.213). Population status for mammals was significantly positively related to proportional funding, but negatively related to critical habitat designation (N = 29; pseudo R^2^ = 0.399). The proportion of recovery objectives attained for plants was significantly positively related for years listed, peer-reviewed information and proportional funding (N = 519; pseudo R^2^ = 0.193).

Species' recovery scores were not significantly related to whether, or how long, CH had been designated. Species with CH designation were not doing better, on average, than those without. The effect size for CH designation remained small and insignificant when analyzed separately for each threat category (habitat loss versus other threats). There was no difference in the average status before and after CH designation (median difference = 0.0). This was also the case for the control group of species without CH designation (median difference = 0.0). These results were the same for both measures of recovery.

The proportion of reporting periods for which a species' status was known was positively related to peer-reviewed scientific information (Fig. 3b) and years listed , and it varied significantly among taxonomic groups (p<0.0001 in all cases; R^2^ = 0.127). For all species, the average proportion of reporting periods for which a species' status was known was 0.68; birds and fish had the highest proportions while plants had the lowest.

## Discussion

Earlier studies have reported statistically detectable associations between the recovery of species listed under the Endangered Species Act and the main tools enabled under the act. In this study, we show that: 1) those effects have not been consistently detectable in earlier work, and 2) the effect sizes are very small. The variation among listed species in two measures of recovery – the number of recovery objectives achieved and the change in species status over time – is, at best, only weakly related to the main tools enabled under the Act. The present study considers more species, more indicators of recovery, and more variables that potentially influence recovery than any earlier study, and we still find only weak effects, or none at all. Results in earlier studies were inconsistent (see Introduction above) probably because, when effect sizes are very small, small differences among data sets (and collinear variables) make parameters estimates highly unstable.

There are two possible interpretations of our data. One must conclude either that the tools provided by the ESA have had only modest impacts on the recovery of ESA-listed species over 18 years (at best), or that data used to assess recovery are too imprecise to show whether the tools have had a substantial effect or not. Either way, strong evidence that the tools provided by ESA are working is lacking. To manage recovery of imperiled species, it is essential to assess the effectiveness of management actions, and to modify them to improve outcomes.

The aggregate evidence (ours, plus earlier studies) regarding the beneficial effects of being listed under the ESA is mixed. The best among the weak predictors of recovery in our study is the number of years a species has been listed (Table 1) which implies some benefit from protection from take and section 7 consultations. Other studies have reported a significant correlation between number of years listed and species status [9], [27]. Taylor et al. [10] found a positive effect of years listed, after accounting for CH designation and recovery plans. In contrast, Ferraro et al. [28] found a *negative* effect of being listed on species status. They compared ESA-listed species to a control group of species from the Nature Serve data base and their study was limited to 135 vertebrate species. They found that listing was only beneficial when combined with high levels of funding. Inconsistent effects probably reflect small absolute effect size and imprecise data.

The aggregate evidence about the effects of recovery plans is also mixed. We observed a positive effect on recovery objectives achieved, but not on species status trends (Table 1). Other studies have observed positive effects of recovery plans when those plans focused on single species and/or had a diversity of authors, but not for multi-species recovery plans [8], [10], [22]. Perhaps the reason we only see an effect of recovery plans in two of our four models is that we did not distinguish between single- and multi-species plans.

The effect of funding on ESA-listed species has been examined in many other studies, but we are the first to examine both absolute funding and funding as a proportion of the estimated amount required for species recovery. We found that recovery was more strongly related to proportional funding than to absolute funding, but the effect was still modest (Table 1). Male and Bean [9] found that recovery was significantly related to annual FWS+NOAA funding. They do not quantify the strength of this relationship; however, all of the variables included in their study explained only 13% of the variation in species' status, including variables such as “risk of extinction” and “recovery potential”, so necessarily the effect of funding was small. Kerkvliet and Langpap [8] found that an additional million dollars in funding decreased the likelihood of a species being listed as extinct by less than 1% and declining by 1.3–1.7%, but that it did not increase the probability of being stable or increasing. Kerkvliet and Langpap's [8] study was limited to vertebrate species with no unknown status reports (i.e., 19% of all listed species), which generally had high funding levels, so their results cannot be applied to listed species in general. Miller et al. [21] looked at funding as a proportion of the amount requested in the species recovery plan that had been received and found that species with higher funding were more likely to be stable or increasing (although, again, they did not specify effect size).

While the detectable effects of funding on recovery may be modest, the amount of information available on ESA-listed species relates more strongly to funding, both in terms of peer-reviewed scientific publications and availability of assessments of recovery status. Mean yearly funding and numbers of publications are strongly correlated (Fig. 3a), and there is a positive relationship between the proportion of known status reports and mean yearly funding (Fig. 3b) and peer-reviewed information (Fig. 3c). This is consistent with the notion that a portion of species funding goes towards research which provides more information on species status. However, even this relationship accounted for only 12% of the variability in available reports.

The aggregate evidence regarding critical habitat suggests that there is no detectable effect. We found that species with CH designation are not doing better than those without it. We tested this both with a general linear model and by looking the difference in average status before and after designation. The studies of Male and Bean [9] and Kerkvliet and Langpap [8] were also consistent with this conclusion. In contrast, Taylor et al. [10], who reported a positive effect of CH designation, looked at two time periods, 1990–1994 and 1997–2002, and tested whether or not species with CH in each period were more likely to be increasing and less likely to be decreasing than those without it. Only two of their four tests were significant. One explained less than 1% of the variation in status, the other explaining less than 10%. We conclude that the relationship between species status and CH is, at best, very weak.

Given that habitat loss is cited as the main threat to imperiled species in the U.S. [29] one would expect CH designation to have a strong positive effect on species status. However, legal designation of CH does not necessarily mean that habitat is protected on the ground, since CH designation applies only to situations involving federal agencies [20]. Suckling and Taylor [17] provide a number of case studies where CH designation was used to provide effective habitat protection. However, for endangered species generally, CH designation that is limited to the actions of federal agencies is apparently insufficient to promote recovery appreciably.

We suspect that the ESA tools we studied may be more effective than our study suggests, but that the species recovery data are grossly inadequate. Species population status data are published in biennial recovery reports to Congress as mandated by the Act. If species status data are available at all, they are qualitative and are relative to a previous recovery report. There are no standards on how status decisions are made, nor are the reports peer reviewed in any way. Many of the status assessments are based on the opinion of FWS staff [22]. Despite this, species status reports have been used in most of the previous assessments of the effectiveness of the ESA [9], [10]. Due to these limitations we used a second measure of species recovery – the number of recovery objectives achieved. But this measure also has severe limitations. The recovery objectives outlined in the recovery reports have been criticized as being arbitrary and not based on science [22], [30].

We have no independent verification of the quality of species status and recovery objective data. The two recovery metrics that we studied are positively correlated (r = 0.49; see also [8], [31]), but for a given recovery objectives achieved score, there is a large amount of variation in species population status, especially for the lower scores (Fig. 4). This suggests that the FWS population status scores are indeed very imprecise indicators of species' recovery status [4]. Accurate, quantitative information on species status is necessary for assessing the ESA and subsequently improving and strengthening it.

**Figure 4:** Relationship between population status and recovery objectives achieved. Scatter plot showing the relationship between change in population status over time and recovery objectives achieved for ESA listed species. Data comes from biennial FWS recovery reports to Congress. Line shows LOWESS smoothing functions with tension = 0.7. N = 1179.

Another criticism of the ESA is that delays in listing at-risk species results in species not being listed until their situation is already critical [4], [32]. Greenwald et al. [32] found that the average time to list a candidate species was 11 years. They note that these delays make recovery very difficult, and in some cases, impossible. Perhaps tools would be more effective if species were listed more quickly.

Despite including more species and more variables than previous studies, we find that species recovery is, at best, only weakly related to the main tools enabled under the Act. We are not suggesting that the Act should be abandoned; there is no way to know what would have been the fate of listed species in the absence of protections offered by the Act. We have no direct evidence to assess whether the Act *per se* is flawed, or the implementation of the Act is flawed (perhaps because of lack of funding), or the data available to assess the implementation are flawed. It is critically important to assess the effectiveness of tools used to promote species recovery; it is therefore also critically important to obtain population status data that are adequate to that task.

## Supporting Information

Dataset S1 **Listing, status, funding, and threat variables for 1251 species listed under the Endangered Species Act prior to 2003.**
(XLSX)
